# Analysis of Winning Experience and Technical Training Effect of Badminton Match Based on BP Neural Network

**DOI:** 10.1155/2022/5295881

**Published:** 2022-02-21

**Authors:** Honglian Song

**Affiliations:** School of Physics Education, Nanjing Forestry University, Nanjing 210037, Jiangsu, China

## Abstract

The success or failure of badminton competition often depends on the training level of technical, physical, tactical, and psychological quality, as well as the competitive ability to comprehensively use these factors in the competition. Aiming at the improvement of the BP neural network algorithm, the improved BP neural network algorithm is used to analyze the multidimensional attributes of the collected data, and the simulation experiment is carried out to find out our competitive advantages and disadvantages. This paper presents a statistical study on the change of service area, the application of service receiving technology, and the treatment of the third stroke technology in the badminton competition. The innovative contribution of this paper is to explore the differences of double service decision-making of badminton at different levels and form a theoretical mechanism analysis system. The research shows that the relationship between active and passive attack and hitting quality has been dealt with in the game. In training, mastering the basic technical movements of badminton is conducive to improving the technical level of badminton.

## 1. Introduction

Badminton is a relatively wide range of sports activities in China. Badminton has been introduced into China from abroad for only a few decades, but the level of badminton in China has been in the leading position in the world [1]. Badminton techniques are characterized by consistency, flexibility, and mutation. Many technical actions are very similar in the preparation process before hitting the ball. Sudden changes in the instant of hitting make the film unexpected [2]. The statistical analysis system of badminton on-the-spot tactics is established by means of sports informatization and BP neural network algorithm to meet the requirements of the development law of badminton sport. At the same time, the establishment of this system can provide information management and tactical decision support services for badminton teams at all levels in China [3]. The game data of badminton were sorted out, and a unified database of smart hairballs was established to solve the problem that the data collection of badminton training games was not timely and comprehensive [4]. It is often necessary to make a prejudgment before the opponent hits the ball or at the moment of the ball. In order to make accurate prediction, it is necessary to be able to observe important prior information related to the opponent's way of hitting the ball and even use the game experience to quickly infer the opponent's way of hitting the ball [5]. The badminton doubles project is faster than the singles project and requires more decision-making speed for badminton games. On this basis, the BP neural network algorithm technology is used to dig deeper into the collected data to find out the weaknesses and advantages of the badminton game [6].

The fast, accurate, ruthless, stable, and changeable technical and tactical characteristics of badminton determine that on the basis of the overall development of physical quality, the badminton match should highlight the special qualities of speed, speed strength (explosive force), and strength endurance [7, 8]. This provides accurate data reference for coaches' on-the-spot command and helps coaches and badminton match timely adjust the strategy and tactics of follow-up matches. This function can change the situation that coaches can only rely on manual records and experience to conduct matches on the field in the past and provide strong support and guarantee for the scientificalization of coaches' on-the-spot command [9]. By analyzing the relationship between the physiological index of the badminton match and the training data, the output problem becomes a nonlinear optimization problem. The adjustment is that the error propagates from the back to the front, so this neural network is also called the BP network [10–12], establishing the scientific analysis and evaluation system of a competitive state, realizing the customization of the scientific training plan on the basis of ensuring the most reasonable physiological and psychological load of the badminton game, and providing technical support for the comprehensive improvement of the competitive state of the badminton match. The competition on the badminton court is not only the competition between the players but also the competition of the coaches, researchers, and other service personnel. Looking at the world of badminton, the general trend of badminton sports technology and tactical development is developing toward comprehensive technology and tactical changes [13].

In order to provide auxiliary support for improving badminton skills and tactics, it is necessary for us to use these past statistical data to discover new useful knowledge [14]. There are many unknown items or attributes in the existing statistics of badminton matches. The rule of the BP neural network is a method specially used to discover the implicit relationship between these data [15]. The connection weight of the neural network is an adjustable parameter, which is equivalent to the particles in the solid material, and the output error of the neural network is equivalent to the energy state of the solid material. The adjustment of the connection weight of the neural network does not necessarily reduce the output error of the neural network [16]. Before the development of the observation form, some experts and some teachers and coaches who have been engaged in badminton teaching and training for many years were interviewed. At the same time, interviews were held on some doubles professional badminton competitions. The content of the interviews provided the basis for the analysis and discussion of this paper [17]. The purpose of improving the use of technology is to use certain technology in the game to make it play a certain role. For example, after gaining the initiative in the backcourt, I want to organize an attack, which is to level the high ball and not to play the high ball. If the opponent is forced to lose the center position, to speed up, the sling and kill technique should not be adopted. Light crane technology [18]was adopted to explore the relevant nature of sports expectations and sports levels in badminton competition scenarios. The differences in decision-making between different levels of badminton games were found through research. The expected advantages of sports experts are mainly reflected in the expected correct rate, and there is no advantage in the expected response [19].

In this paper, we put forward an algorithm of the BP neural network, which is an algorithm that should be analyzed and constructed for the winning experience and technical training effect of badminton matches.

In summary, our contributions are as follows:

1. This algorithm is a new algorithm based on a BP neural network, which aims at the difficult problem of winning experience and technical training effect in badminton matches
2. This algorithm is widely applicable in the environment of the BP neural network, and it should be analyzed and constructed for the winning experience and technical training effect of badminton matches
3. This algorithm has higher recognition, higher accuracy, and better results

## 2. Related Work

Gajhede-Knudsen et al. conducted a series of three experiments in 2013 to screen the video of badminton matches in time and space and to explore the ability of judging the batting mode in different levels of badminton matches. The results showed that the judgment ability of novice badminton game decreased significantly after the amount of information of batting in the video was reduced [20]. In the same year, Abian-Vicen et al. studied the difference in prejudging ability of receiving badminton matches in different levels through space blocking technology. In the test, the racquet, upper limbs, and shoulder-chest (torso) parts of the player in the video were separately shaded. It was found that the accuracy of the prejudgment of the badminton game under the shielding condition decreased, and there was no difference in the response when shielding the different parts [21].

Huang et al. pointed out in 2014 that oral report is also a kind of “data”. The oral report can compensate for the internal thinking process and psychological changes of subjects in simulated situations when they make decisions. These data cannot be measured by eye trackers and image stereotyping technology [22]. In 2015, Phomsoupha et al. used the oral report method to study the differences in problem representation and thinking characteristics of different levels of badminton games. It was found that the expert's thinking process mainly adopts the “top-down” processing method. Experts have more general concepts, conditional concepts, and action concepts in problem representation. They can make decision-making training on badminton games by changing the video playback speed of the hairball game. It is found that speeding up the video speed can more realistically simulate the real game situation. It is feasible to use this method to make decision-making intervention training for badminton games [23].

## 3. Materials and Methods

Competition is in a certain time, space, in the fierce offensive and defensive confrontation conditions, and it will inevitably cause a strong physiological and psychological burden to badminton competition. Badminton matches must meet the requirements of the competition and improve the competitiveness. Serving is the only technique that is not restricted by the opponent. The server can serve the ball with a different speed and landing point at will. Therefore, the server generally possesses initiative. In the competition, whether it is a general level badminton match or a world-class badminton match, it is particularly important to receive the other side's service. Because it is difficult to define the weights of technical means in badminton with specific numerical values, when we design the BP neural network algorithm model, we define the types of project constraints as the first kind of constraints, that is, to constrain the batting area and the items of technical parameters, in order to find the rules between gains and losses. The change in the connection weight of the neural network can be combined with the backpropagation error and random number, and the connection weight can be adjusted according to the criteria. If the output error decreases, the adjustment of the connection weight will be accepted; if the change in the connection weight of the neural network increases the output error, the adjustment of the connection weight will be accepted with a certain probability. The data conversion of the BP neural network is shown in Table 1, and the BP neural network model is shown in Figure 1. There is no interaction between the test phase and the intervention mode, and the decision-making response of the testee is not affected by the test phase and the training mode. At the same time, the daily training situation is stored in the mobile terminal in real time, the simple and intuitive data display can be performed and uploaded to the server-side database, and the server side extracts and integrates the game data documents compiled by the coach.

When the opponent returns, he can accurately judge the direction and landing point of the ball, appear there in time, and take the initiative to control the situation of the game. In addition, we should also make an article on the action, make changes in the moment of the action, and try to conceal the action. To interfere with the other party's judgment, cause the other party's judgment errors, so that the other side cannot defend. If the curvature of the arc is large, the speed of the ball coming will be slow, and if the curvature of the relative arc is small, the speed of the ball coming will be fast. The direction of the ball can also be seen as a diagonal line or a straight line. Generally speaking, the coming ball is slanted more slowly than the straight coming ball. The second is to judge the route and the landing point of the service. The landing point is an important factor affecting the batting quality. Develop sensitivity and flexibility in specific physical fitness through ligament pulling and various response abilities. When coaches analyze, they also waste a lot of time. The improvement of the BP neural network algorithm for the above problems can improve the efficiency of the system's on-site decision-making and has important application value for adapting to fast-paced international events. After research and analysis, physical fitness training promotes the learning and improvement of badminton skills. Therefore, the technical quality of the badminton competition is evaluated to help the badminton match improve and adjust the tactics in time and improve the scoring rate. It can also remotely store data on the server-side database, summarizing the relevant rules of the scoring rules and technical and tactical quality of each badminton match.

The name classification of badminton technology has its own different viewpoints and annotations. There are many kinds of categorization of badminton receiving and serving technology, but for the need of research, categorization parameters of badminton receiving and serving are shown in Table 2 and Figure 2.

Through boring physical fitness training, but with a variety of training methods, physical fitness training will be integrated into the special training of badminton competition. In this way, the badminton match in their favorite sports training at the same time carried out special physical quality training, so that the badminton game's special technical level has been improved. The badminton's core strength training can significantly improve the speed of badminton movement. A back-throwing solid ball is used to evaluate the upper limb strength, but its movement structure is beyond the equipment and the final whip action. Badminton, whether killing or high-altitude ball, requires coordination of upper and lower limbs, and the whole body strength gathers at one point. In daily training and competitions, the coaches mainly rely on on-site observation and experience to conduct training quality evaluation and on-the-spot commands for badminton games, lacking accurate and comprehensive data support. From the point of view of data collection, it is not intuitive to manually record on paper by the coach. In the preprocessing module of the experimental data, we discretize the numerical attributes according to the standards provided by the national badminton team. Secondly, the hitting point of the ball in the badminton game cannot be over the waist, and the whole ball head needs to be significantly lower than the whole. Hold the hand. In the end, the player's service must be swung forward until the ball is hit; that is, there are no restrictions such as fake movements, so the ball from the badminton game cannot be counted as the first attack. Therefore, it will be less likely that the receiving and receiving sides will be passive.

Combining badminton skills with physical fitness training is the application factor of this experiment. The purpose is to infiltrate physical fitness training into badminton's special teaching. The endurance quality training methods are shown in Table 3 and Figure 3. The speed quality training methods are shown in Table 4 and Figure 4.

## 4. Result Analysis and Discussion

Under such circumstances, we can cultivate the fighting spirit and perseverance of badminton matches and also require that the special badminton matches must be highly focused on multiball training. In addition, multiball training in badminton technical movements can help badminton matches correct wrong technical movements and improve their technical level. To create specific teaching scenarios in line with physical education teaching, service badminton matches, when serving, will take into account the issue of service tactics. Therefore, when serving, the server will achieve a combination of hard and soft (there are changes in the batting movements when serving). The rhythm of service includes tight and loose, a combination of lengths (a combination of inner and outer corners in the latter half and inner and outer corners in the former half), and a combination of straight line and diagonal. Guide badminton matches to trigger emotional experiences through personal practice and then help them accurately understand the content of physical education. Regardless of the actual needs, they reveal the network of data between these data. If the data to be analyzed take into account the actual needs in the value, it is divided into different levels, and it is easy to accept the deterioration solution so that the connection right adjustment range is large. It is possible that the final result is not as good as the result at some point in the middle. Then reveal the relevance of the connection between these data. Save the generated data to an intermediate database. In addition, since the data in the integrated database mainly provides the query function, the introduction of the intermediate library can separate the data used by the BP neural network algorithm from the original data and avoid the influence of redundancy and inconsistent data generated in the data processing process on the information query.

The main techniques of badminton (forehand serve, forehand strike, and forehand smash) are evaluated and tested to meet the technical standards. The overall technical evaluation results of badminton matches and multiball training teams' badminton matches are shown in Table 5 and Figure 5.

In view of the fact that there are not many kinds of statistical data items for badminton techniques and tactics, we can introduce a threshold value through the BP neural network, which combines the advantages and characteristics of this algorithm:

(1) $$\begin{array}{c} \frac{\text{d}i}{\text{d}t}=\lambda \cdot s\left(t\right)\cdot i\left(t\right). \end{array}$$

A constraint is the one that can be converted to

(2) $$\begin{array}{c} s\left(t\right)+i\left(t\right)=1. \end{array}$$

That is to say, reducing the number of candidate item sets can effectively improve the efficiency of the algorithm:

(3) $$\begin{array}{c} i\left(t\right)=\frac{1}{1+\left(1/i_{0}-1\right)\cdot e^{-\lambda t}} \end{array}$$

Then the new state will accept the change as an “important” state:

(4) $$\begin{array}{c} t_{\max}=\frac{1}{\lambda }\ln\left(\frac{1}{i_{0}}-1\right). \end{array}$$

Then accept the change of the connection weight; otherwise, keep the original connection weight. The probability that the connection weight is modified is defined as

(5) $$\begin{array}{c} dR_{t}=\chi \cdot a\left(t\right)\cdot dt+\delta \cdot a\left(t\right)\cdot dw_{t}\frac{n!}{r!\left(n-r\right)!} \end{array}$$

When the connection right accepts the inverse correction, the probability is small, according to the formula:

(6) $$\begin{array}{c} dR_{t}^{\pi }=\xi \cdot a_{\pi }\left(t\right)dt+\zeta \cdot a_{\pi }\left(t\right)\cdot dw_{t}-dU_{t}^{\pi }. \end{array}$$

The connection weight is adjusted inversely with a certain probability, so the global optimal value can be found for the overall convergence problem:

(7) $$\begin{array}{c} H\left(x,\pi \right)=E\left[\left(\int_{0}^{\pi }e^{-cs}\cdot \text{d}L_{s}^{\pi }\right)\right]. \end{array}$$

That is, each connection weight component is added with a “random number,” which is generated by the product of backpropagation error and random number:

(8) $$\begin{array}{c} H\left(x,\pi_{b0}\right)=\underset{\pi \in \Pi_{0}}{\sup}H\left(x,\pi \right),\\ V\left(x\right)=\underset{b}{\sup}\left\{V\left(x,b\right)\right\}. \end{array}$$

Calculate the output error of the neural network before and after the change of the connection weight:

(9) $$\begin{array}{c} R_{t}^{\pi *}=x+\int_{0}^{t}\xi \cdot a\left(R_{s}^{\pi *}\right)\cdot \text{d}s+\int_{0}^{t}\zeta \cdot a\left(R_{s}^{\pi *}\right)\cdot \text{d}w_{s}-U_{t}^{\pi *}. \end{array}$$

If the neural network output error meets the requirements, the training learning ends:

(10) $$\begin{array}{c} P_{i}=F\left(Y_{i}\right)=\frac{e^{Y_{i}}}{1+e^{Y_{i}}}. \end{array}$$

Sometimes jump from the best to other points and get the true optimal value by comparison.

(11) $$\begin{array}{c} Y_{i}=\alpha +\sum_{j=1}^{k}\beta_{j}\cdot X_{ji}. \end{array}$$

Improve the level of a special quality of badminton matches, but in the proportion of training, according to the difference in physical quality and technical characteristics of the training object, there will be a different proportion. In addition, core strength training can effectively reduce the incidence of sports injuries, improve the transmission of strength, and promote the development of special sensitive qualities. The level of physical fitness has been improved; on the other hand, they firmly grasp the badminton technology. Serving well or badly can directly affect the players to strive for initiative or the players are in a passive situation. Master the serving technique well, and choose the serving method which is advantageous to the attack according to the opponent's merits and demerits in the match, to force the opponent to be caught unprepared or passive, so as to achieve the goal of winning the initiative score. Force the opponent to expose his patience weakness, and wait for an opportunity to fight back; to deal with tall, turn, and footwork is not good, but killing the opponent with good Internet, first of all, we should pay attention to the advantage of killing the opponent with Internet, when the opponent uses killing the Internet. We should not only be able to defend it but also destroy its advantages by hooking diagonal balls and seizing their weaknesses of inadequate rotation and gait. The classification of the receiving server is divided into the front ball and the backfield. The receiving service statistics are shown in Figure 6. In this paper, the observation data are organized into the starting point and the landing point of the badminton on the simulation field of the system. The system will automatically judge the record player, the selection area, and other information according to the selection and automatically list the score type, technology type, etc. For selection, the specific score data of the two badminton games will also be displayed dynamically. They often participate in extracurricular badminton activities and use the physical fitness practice methods used in teaching. This practice method is effective.

Especially when the competition is fiercest, usually due to lack of physical strength, players will show deformations in technical movements and increase in active errors, slow down obviously, and be limited by the other side, which will lead to the loss of the game. Physical strength has always been a common problem in badminton competitions. Physical fitness training is the basis of all training. Strengthening the training of physical fitness is to accumulate energy, and practicing sports skills is to reduce energy consumption. However, whether it is in physical fitness training or in sports skills training to reduce energy consumption, both of them directly affect badminton's sports level. Therefore, physical fitness and badminton skills are complementary. The parameters are attenuation coefficients, which can control the optimization speed of connection weight. The larger the value is, the slower the attenuation of the sample is, and the larger the search range of the connection weight is. The value is small, the attenuation of the sample is faster, but the search range is reduced, and the iterative change of BP neural network parameters is shown in Figure 7. Various data collected by the mobile terminal can be uploaded to the server and sent to the back-end database. On the background server side, it manages auxiliary information such as personnel information and technical information. At the same time, coaches can view and edit the badminton tournament week training program and the day training program on the mobile side. Import and count past technical and tactical documents and establish a comprehensive information platform. In addition, it can be seen from the high-ranking event that the opponent has a high success rate when using the backhand attack, which indicates that the player has some shortcomings in the route of the backhand ball, which can be targeted. The training program provides help in decision making.

## 5. Conclusion

In this paper, the application of the BP neural network algorithm in badminton competition winning experience and the technical special training effect are analyzed. If we want to win the game, we should be able to take the initiative in attack-defense conversion and score in multishot under the premise of dealing with the reception and delivery. Therefore, in training, we should strengthen training not only in technology, but also in physical endurance, strength, and other qualities. In badminton matches, all distractions and interference should be eliminated and attention should be paid to the rational use of techniques and tactics. The combination of live practice and video decision-making training is an effective way to improve the decision-making ability of new badminton players. The decision-making ability of new badminton players through decision-making training has been significantly improved compared with those without training. As long as you insist on doing this every time, you will definitely play the game further and welcome more victories. At the same time, it is necessary to carry out the analysis conclusions and the feedback from the coaches and further modify the parameters of the data conversion model to make it more suitable for the characteristics of the badminton sport itself. Combine body function action screening results with areas of insufficient functionality. Carry out the correct action guidance, master the real core area stability sensory system, and then experience the core area power elements and improve the body movement function level.

## Figures and Tables

**Figure 1:** BP neural network model.

**Figure 2:** Technical parameters of receiving and serving in badminton doubles.

**Figure 3:** Endurance quality training.

**Figure 4:** Speed quality training.

**Figure 5:** Analysis of badminton major technical test achievements.

**Figure 6:** Statistics of receiving and serving techniques.

**Figure 7:** Iterative variation of BP network parameters.

**Table 1:** Data conversion of the BP neural network.

	Constraint	Transformation
Dimensionality reduction	16.90	15.46
Null value processing	15.73	16.72

**Table 2:** Technical parameters of receiving and serving in badminton doubles.

	Judge	Influence
Front-court receiving and serving techniques	3.64	2.94
Backcourt receiving technology	3.05	2.58

**Table 3:** Endurance quality training.

	Load capacity	Decision number
Speed endurance	23.64	19.09
Aerobic endurance	26.82	18.33

**Table 4:** Speed quality training.

	Load capacity	Decision number
Action speed	20.64	15.42
Reaction rate	21.30	16.50

**Table 5:** Analysis of badminton major technical testachievements.

	Average	Standard deviation
Serve	84	0.64
Batting	71	0.92
Smash	68	0.81

## Data Availability

The data used to support the findings of this study are included within the article.

## References

[1] Arora M., Shetty S. H., Khedekar R. G., Kale S. (2015). Over half of badminton players suffer from shoulder pain: is impingement to blame?. *Journal of Arthroscopy and Joint Surgery*.

[2] Loureiro L. d. F. B., De Freitas P. B. (2016). Development of an agility test for badminton players and assessment of its validity and test-retest reliability. *International Journal of Sports Physiology and Performance*.

[3] Lin C.-F., Hua S.-H., Huang M.-T., Lee H.-H., Liao J.-C. (2015). Biomechanical analysis of knee and trunk in badminton players with and without knee pain during backhand diagonal lunges. *Journal of Sports Sciences*.

[4] Ebrahim J., Ali M., Maryam H., Musavian R., Abbasi E. (2013). Comparison of blue-yellow opponent color contrast sensitivity function between female badminton players and non-athletes. *Asian Journal of Sports Medicine*.

[5] Abian P., Del Coso J., Salinero J. J. (2015). The ingestion of a caffeinated energy drink improves jump performance and activity patterns in elite badminton players. *Journal of Sports Sciences*.

[6] Park J., Lee Y. H., Kong I. D. (2017). Ultrasonographicchangesof upperextremitytendonsinrecreationalbadmintonplayers: Theeffectofhanddominanceandcomparisonwithclinicalfindings. *British Journal of Sports Medicine*.

[7] Jafari A., Golami M., Mabani M., Mabani M. (2014). The prevalence and causes of sport injuries in well-trained badminton players of Iran. *International Journal of Sciences: Basic and Applied Research*.

[8] de França Bahia Loureiro L., Dias M. O. C., Cremasco F. C., da Silva M. G., de Freitas P. B. (2017). Assessment of specificity of the badcampagility test for badminton players. *Journal of Human Kinetics*.

[9] Hülsdünker T., Strüder H. K., Mierau A. (2016). Neural correlates of expert visuomotorperformance in badminton players. *Medicine & Science in Sports & Exercise*.

[10] Hülsdünker T., Strüder H. K., Mierau A. (2017). Visual but not motor processes predict simple visuomotor reaction time of badminton players. *European Journal of Sport Science*.

[11] Bisschoff C. A., Coetzee B., Esco M. R. (2018). Heart rate variability and recovery as predictors of elite, African, male badminton players’ performance levels. *International Journal of Performance Analysis in Sport*.

[12] Linnebjerg C., Zebis M., Merete M., Vollaard N. (2017). Shoulder functionandshouldercomplaintsinDanishelitebadmintonplayers. *British Journal of Sports Medicine*.

[13] Khan M. J., Giasuddin A. S., Khalil M. I. (2015). Risk factors of tendo-achillesinjury in football, cricket and badminton players at Dhaka, Bangladesh. *Bangladesh Medical Research Council Bulletin*.

[14] Abián P., Del Coso J., Salinero J. J. (2016). Muscle damage produced during a simulated badminton match in competitive male players. *Research in Sports Medicine (Print)*.

[15] Abian-Vicen J., Castanedo A., Abian P., Gonzalez-Millan C., Salinero J. J., Coso J. D. (2014). Influence of successive badminton matches on muscle strength, power, and body-fluid balance in elite players. *International Journal of Sports Physiology and Performance*.

[16] Fuchs M., Faude O., Wegmann M., Meyer T. (2014). Critical evaluation of a badminton-specific endurance test. *International Journal of Sports Physiology and Performance*.

[17] Bisschoff C. A., Coetzee B., Esco M. R. (2016). Relationship between autonomic markers of heart rate and subjective indicators of recovery status in male, elite badminton players. *Journal of Sports Science &Medicine*.

[18] Zhu Q. (2013). Perceiving the affordance of string tension for power strokes in badminton: Expertise allows effective use of all string tensions. *Journal of Sports Sciences*.

[19] Cruz A. B., Kim H. D (2017). Leadership preferences of adolescent players in sport: Influence of coach gender. *Journal of Sports Science &Medicine*.

[20] Gajhede-Knudsen M., Ekstrand J., Magnusson H., Maffulli N. (2013). Recurrence of Achilles tendon injuries in elite male football players is more common after early return to play: An 11-year follow-up of the UEFA Champions League injury study. *British Journal of Sports Medicine*.

[21] Abian-Vicen J., Castanedo A., Abian P., Sampedro J. (2013). Temporal and notational comparison of badminton matches between men’s singles and women’s singles. *International Journal of Performance Analysis in Sport*.

[22] Huang M.-T., Lee H.-H., Lin C.-F., Tsai Y.-J., Liao J.-C. (2014). How does knee pain affect trunk and knee motion during badminton forehand lunges?. *Journal of Sports Sciences*.

[23] Phomsoupha M., Laffaye G. (2015). The science of badminton: game characteristics, anthropometry, physiology, visual fitness and biomechanics. *Sports Medicine*.

